# Improved Fuzzy C-Means Clustering Algorithm-Based Dynamic Contrast-Enhanced Magnetic Resonance Imaging Features in the Diagnosis of Invasive Breast Carcinoma before and after Menopause

**DOI:** 10.1155/2022/2917844

**Published:** 2022-06-18

**Authors:** Li Mei, Kaixiang Wang, Yongjian Gu

**Affiliations:** ^1^Department of Imaging, Wujin Hospital Affiliated with Jiangsu University, Changzhou 213003, China; ^2^Department of Imaging, The Wujin Clinical College of Xuzhou Medical University, Changzhou 213003, China

## Abstract

The application effect of dynamic contrast-enhanced magnetic resonance imaging (DCE-MRI) based on the improved fuzzy C-mean clustering (GA-PFCM) algorithm in analyzing premenopausal and postmenopausal invasive breast carcinoma was discussed. 159 patients with breast carcinoma were selected and divided into the postmenopausal group (71 patients) and the premenopausal group (88 patients) according to their menstrual status. The magnetic resonance images of the two groups were processed and analyzed using GA-PFCM algorithm, and the imaging characteristics and relevant parameters of DCE-MRI examination of the two groups were analyzed. Besides, the sensitivity, specificity, and accuracy of the diagnosis of invasive breast carcinoma by DCE-MRI examination were investigated. The results showed that the percentage of patients with lobulated lumps, patients with burrs on lesion edge, and patients with uniformly enhanced tumors in the premenopausal group was larger than that in the postmenopausal group (*P* < 0.05). In the postmenopausal group, TCI of 33 patients was shown as platform curves, and that of 34 patients was shown as outflow curves. In the premenopausal group, TCI of 39 patients was shown as platform curves, and that of 41 patients was shown as outflow curves with a high proportion. The number of patients with peak height time ranging between 130 s and 260 s and of patients with early signal enhancement rate ranging between 100% and 200% was large. In contrast, the number of patients with ADC value higher than 1.2 × 10^−3^ was the least. In this research, there were 128 patients with positive invasive breast carcinoma and 31 with negative invasive breast carcinoma by pathological examination. Based on DCE-MRI examination, there were 121 patients with positive invasive breast carcinoma and 38 with negative invasive breast carcinoma. The sensitivity, specificity, and accuracy of invasive breast carcinoma by DCE-MRI were 91.41%, 87.1%, and 90.57%, respectively. In addition, the positive and negative predictive values reached 96.69% and 71.05%, respectively. In summary, GA-PFCM algorithm can be applied in the processing and segmentation of DCE-MRI images, and DCE-MRI could better diagnose invasive breast carcinoma with positive guiding value.

## 1. Introduction

In recent years, the incidence of breast carcinoma increases significantly [1]. Breast carcinoma is a malignant tumor that occurs in breast ducts and epithelium and a highly heterogeneous cancer [2]. Breast carcinoma is divided into several subtypes. Previously, tumor lymph node metastasis (TNM) staging and histologic classification were commonly used to determine the prognosis of breast carcinoma and predict the probability of its recurrence and metastasis. However, immunohistochemical test becomes a common method for predicting the clinical course of disease and is correlated with specific gene expression patterns in recent years [3]. The risk of suffering from the disease among the relatives of patients with breast carcinoma triples [4]. Age, parity, family history, and menstruation status affect the incidence of breast carcinoma. Breast carcinoma occurs among middle-aged and elderly women most frequently [5]. Environmental pollution and food safety have a significant impact on the prevalence of breast carcinoma among women. Menstruation is formed after hormones secreted by ovary act on endometrium, and whether menstruation is normal is closely related to the level of hormones in the body. Breast carcinoma is a hormone-dependent tumor. When menstruation becomes abnormal, estrogen, progestogen, and androgen disorders occur, which increases the incidence of breast carcinoma [6]. Invasive breast carcinoma is the commonest type among breast carcinoma, accounting for around 80% of all breast carcinoma [7]. The cells in invasive breast carcinoma break through the basement membrane of the ductal wall with poor prognosis.

Breast magnetic resonance imaging (MRI) becomes an essential method of assessing breast carcinoma lesions, detecting tumor recurrence, and evaluating therapeutic effect on breast carcinoma. It can be used for the clinical assessment of postoperative tumor staging and residual disease after treatment and shows positive application value [8]. Dynamic contrast-enhanced magnetic resonance imaging (DCE-MRI) plays an important role in the diagnosis and prediction of breast carcinoma. It is featured with high clinical application value and high resolution. A large amount of contrast agent in cancer cells rapidly accumulates in the extravascular-extracellular space. MRI reflects the biological information about cancer carcinoma through hemodynamic parameters to generate the corresponding imaging parameters, which can analyze tumors quantitatively [9]. Fuzzy C-means clustering (FCM) algorithm is a method that can realize automatic classification of samples with simple operation and strong local search capacity [10]. Traditional FCM algorithms only take into account the distance from data points to each clustering center without considering the influences of initial clustering center on segmentation results. As a result, inaccurate segmentation often occurs, which reduces algorithm performance [11]. GA-PFCM algorithm can improve the accuracy of cluster center results and diagnostic efficiency as well as accuracy and has positive application values in the determination of tumor types.

Based on GA-PFCM algorithm, DCE-MRI imaging feature analysis was performed among patients with breast carcinoma before and after menopause. Besides, the imaging features and relevant parameters of DCE-MRI examination of patients with breast carcinoma in the two groups were investigated, and the sensitivity, specificity, and accuracy of the diagnosis of invasive breast carcinoma by DCE-MRI examination were discussed to provide clinical guidance on the processing and analysis of MRI of patients with breast carcinoma and reference for the diagnosis and prediction of breast carcinoma.

## 2. Materials and Methods

### 2.1. Research Objects

A total of 159 patients with breast carcinoma treated at our hospital between June 2018 and December 2021 were selected as the research objects. Patients were divided into two groups according to their menstrual conditions. In the postmenopausal group, there were 71 female patients aged between 55 and 92 with the average of 67.23 ± 7.26. In the premenopausal group, there were 88 female patients aged between 29 and 55 with the average of 36.27 ± 6.79. Among all the included patients, there were totally 128 cases with invasive breast carcinoma and 31 with noninvasive breast carcinoma. The included research objects received DCE-MRI examination and pathological examination to analyze the imaging features and diagnostic effects of DCE-MRI examination for the patients in the two groups. This research had been approved by ethics committee of hospital.

Inclusion criteria are as follows: patients with complete medical records and imaging data; patients without contraindications to MRI examination, severe cardiopulmonary diseases, liver and kidney dysfunction, and ferromagnetic foreign body; patients without undergoing biopsy, surgery, chemotherapy, radiotherapy, and other invasive diagnosis or treatment; and patients diagnosed with breast carcinoma by surgical pathology.

Exclusion criteria are as follows: patients with combined significant organ diseases; patients with central nervous system diseases, endocrine system diseases, and other severe physical diseases; pregnant or lactating women; and patients unwilling to participate in the study.

### 2.2. Magnetic Resonance Examination

GE750w MRI system was used for all research objects, and multichannel phased array breast coil was used. Scan slice thickness should be equal to or less than 3 mm, and interlamellar spacing needed to be 0 mm. During the examination, patients were instructed to take prone position to make both breasts hang naturally in the groove of special breast coil with nipples at the lowest point. Scanning sequence was as follows: axial short recovery time reversal recovery magnetization preparation spin echo pressure T2W1 sequence, transverse three-dimensional fast small angle excitation gradient echo imaging T1W1 sequence, horizontal-axis single excitation spin echo DWI imaging sequence with autonomous shimming and frequency as well as fat suppression technique, and axial fast small angle excitation three-dimensional dynamic imaging fat suppression T1W1 sequence.

### 2.3. Serum Tumor Marker Examination

5 mL patients' venous blood was extracted and centrifuged at 3000 r/min for 10 minutes. Electrochemiluminescence method was adopted to detect serum carcinoma embryonic antigen (CEA)\tissue polypeptide specific antigen (TPS) and CA153 levels.

### 2.4. Steps and Processes of GA-PFCM Algorithm

Float-point encoding was adopted, and each individual was expressed by the floating-point number of *a* × *b*. *a* referred to the number of clusters, and *b* represented data dimension.

Initial population was generated randomly. 3 samples were assigned randomly to 1 class, and their average value was taken as the initial value, which was performed for *n* times.

It was assumed that the image contained *m* points, and the gray scale of the image was divided into *x* classes. *w* denoted fuzzy exponents. The expression of the changed fuzzy clustering target function was shown in equation (1). *u*_*ik*_ represented the dependence level of the *k*th pixel to the *i*th class. *d*_*ik*_^2^ referred to the standard Euclidean distance from the *k*th pixel to the *i*th cluster. *P*_*ik*_ denoted the spatial neighborhood information of the pixel expressed by Markov random fields. *σ* meant constraint coefficient.

(1) $$\begin{array}{c} A\left(U,V\right)=\overset{x}{\underset{i=1}{\sum }}\overset{m}{\underset{k=1}{\sum }}{u_{ik}}^{w}{d_{ik}}^{2}+\sigma \overset{x}{\underset{i=1}{\sum }}\overset{m}{\underset{k=1}{\sum }}{u_{ik}}^{w}{\left(1-P_{ik}\right)}^{w}. \end{array}$$

Fitness was utilized to assess the quality of breast carcinoma images. In most cases, the reciprocal of target function of the optimized FCM algorithm was set as fitness. The calculation method of fitness was expressed as follows:

(2) $$\begin{array}{c} B\left(U,V\right)=\frac{1}{A\left(U,V\right)}. \end{array}$$

Genetic operator was calculated. After selection, chiasma, and mutation, the optimal population was selected.

Whether the termination condition was met was determined. If it was met, the initial clustering center was output; otherwise, the initial population continued to be generated.

The images to be segmented were input, and the initial value was determined by GA. According to PFCM algorithm, images were segmented. When it reached the set threshold or maximum iterations, the iteration of the algorithm was terminated. Next, the pixels were divided, and the image pixels were categorized according to the maximum value of membership. In addition, the gray scale of pixels was updated, and the segmented images were output.

The specific procedures of GA-PFCM are shown in Figure 1. The algorithm could improve image quality and image segmentation effect and assess and diagnose disease better.

### 2.5. Observation Indexes

The general data on the patients in the two groups were summarized, including gender, age, whether they were at climacteric period, breast types, and levels.

The clustering effects of FCM algorithm and GA-PFCM algorithm were compared. The assessment indexes included separation coefficient, separation entropy, and firming and separation effects. The calculation method of separation coefficient was displayed in equation (3), that of separation entropy was shown in equation (4), and that of firming and separation effects were presented in equation (5). *A* (*a*_1_, *a*_2_, ⋯, *a*_*n*_) represented feature space, *k* denoted feature type, and the cluster center of the *x*th type was expressed by *v*_*w*_ ∈ *Rs*. Any feature point *a*_*q*_ ∈ *R*^*s*^ belonged to the membership of the *x*th type *u*_*qw*_.

(3) $$\begin{array}{c} F\left(U,k\right)=\frac{1}{n}\overset{n}{\underset{q=1}{\sum }}\overset{k}{\underset{w=1}{\sum }}{\left(U_{qw}\right)}^{2}, \end{array}$$

(4) $$\begin{array}{c} H\left(U,k\right)=-\frac{1}{n}\overset{n}{\underset{q=1}{\sum }}\overset{k}{\underset{w=1}{\sum }}U_{qw}\log\left(U_{qw}\right), \end{array}$$

(5) $$\begin{array}{c} S\left(U,k\right)=\frac{1/n\sum_{q=1}^{n}\sum_{w=1}^{k}{\left(U_{qw}\right)}^{2}{\left\|a_{q}-v_{w}\right\|}^{2}}{\underset{qw}{\min}{\left\|a_{q}-v_{w}\right\|}^{2}}. \end{array}$$

Breast carcinoma DCE-MRI coefficients of the patients in the two groups were analyzed, mainly including time intensity curve (TIC) types, peak height time, early signal enhancement rate, and apparent diffusion coefficient (ADC) values.

The number of the patients who were negative and positive in DCE-MRI examination and pathological examination was counted, and the diagnostic effects of DCE-MRI examination on invasive breast carcinoma were calculated, including sensitivity, specificity, accuracy, positive predictive value, and negative predictive value. The calculation method of sensitivity was shown in equation (3). The calculation method of specificity was expressed by equation (4). The calculation method of accuracy was displayed in equation (5). The calculation method of positive predictive value was shown in equation (6). The calculation method of negative predictive value was expressed by equation (7). PB referred to the number of the patients with negative invasive breast carcinoma in pathological examination. PM denoted the number of the patients with positive invasive breast carcinoma in pathological examination. YDB represented the number of the patients with negative invasive breast carcinoma and negative pathology in DCE-MRI examination. YDM referred to the number of the patients with positive invasive breast carcinoma and positive pathology in DCE-MRI examination. DB denoted the number of the patients with negative invasive breast carcinoma in DCE-MRI examination. DM represented the number of the patients with positive invasive breast carcinoma in DCE-MRI examination.

(6) $$\begin{array}{c} \text{Sensitivity}=\frac{\text{DM}}{\text{PM}}, \end{array}$$

(7) $$\begin{array}{c} \text{Specificity}=\frac{\text{DB}}{\text{PB}}, \end{array}$$

(8) $$\begin{array}{c} \text{Accuracy}=\frac{\text{DM}+\text{DB}}{\text{PB}+\text{PM}}, \end{array}$$

(9) $$\begin{array}{c} \text{Positive predictive value}=\frac{\text{DM}}{\text{YDM}}, \end{array}$$

(10) $$\begin{array}{c} \text{Negative predictive value}=\frac{\text{DB}}{\text{YDB}}. \end{array}$$

### 2.6. Statistical Methods

SPSS 20.0 was adopted for data statistics and analysis using *t*-test. Percentage was used to represent enumeration data. *P* < 0.05 indicated that the differences showed significant statistical meaning.

## 3. Results

### 3.1. Comparison of the Number of Patients with Different Levels of Breast Carcinoma

The comparison of breast carcinoma levels between the two groups is shown in Figure 2. It was found out that there were 41 patients with level 4b (46.59%), 38 patients with level 4c (43.18%), and 9 patients with level 5 (10.23%) in the premenopausal group. In the postmenopausal group, there were 22 patients with level 4b (30.99%), 31 patients with level 4c (43.66%), and 18 patients with level 5 (25.35%). Obviously, the proportion of patients with level 5 in the postmenopausal group was relatively higher.

### 3.2. DCE-MRI Imaging Features of Patients with Breast Carcinoma

DCE-MRI imaging features of the following 2 patients with breast carcinoma were displayed below. In Figure 3(a), DCE-MRI imaging features of a female patient aged 39 were displayed, including breast carcinoma lumps and burr lobules. In Figure 3(b), DCE-MRI imaging features of a female patient aged 42 were displayed, which was annular enhancement on the edge of breast carcinoma lump.

### 3.3. Comparison of Clustering Effects of Two Algorithms

The comparison of the clustering effects of the two algorithms is shown in Figure 4.  Figure 4(a) represents the separation coefficient, Figure 4(b) denotes the separation entropy, and Figure 4(c) refers to the firming and separation effects. It was found out that GA-PFCM had higher separation coefficient and lower separation entropy as well as firming and separation effect values and better clustering effect than FCM algorithm.

### 3.4. Comparison of Lump Features of Patients with Breast Carcinoma between Two Groups by DCE-MRI Examination

Lump features of breast carcinoma in the two groups by DCE-MRI examination are shown in Figure 5. There were 42 patients with lobular lumps in the premenopausal group and 32 with lobular lumps in the postmenopausal group, and there were 46 patients without lobular lumps in the premenopausal group and 39 without lobular lumps in the postmenopausal group. Besides, there were 36 patients with burrs on lesion edge in the premenopausal group and 25 with burrs on lesion edge in the postmenopausal group. There were 52 patients without burrs on lesion edge in the premenopausal group and 46 without burrs on lesion edge in the postmenopausal group. The number of patients with annular enhanced lumps in the premenopausal and postmenopausal groups reached 51 and 46, respectively. There were 22 patients with inhomogeneous lumps in the premenopausal group and 18 patients with inhomogeneous lumps in the postmenopausal group. In addition, the number of patients with uniformly enhanced lumps in the premenopausal and postmenopausal groups amounted to 15 and 7, respectively. The above results revealed that the proportions of patients with lobular lumps, burrs on lesion edge, and uniformly enhanced lumps in premenopausal group were all higher than those in the postmenopausal group (*P* < 0.05).

### 3.5. Comparison of DCE-MRI Examination Parameters of Patients with Breast Carcinoma

The comparison of breast DCE-MRI examination parameters between the two groups is illustrated in Figure 6.  Figure 6(a) shows the types of TIC curves, Figure 6(b) displays the peak height time, Figure 6(c) illustrates the early signal enhancement, and Figure 6(d) presents the ADC values. It was found out that there were 33 patients with TCI shown as platform curves and 34 with TCI shown as outflow curves in the postmenopausal group. In the premenopausal group, there were 39 patients with TCI shown as platform curves and 41 with TCI shown as outflow curves. The number of patients in the premenopausal group was greater than that in the postmenopausal group. There were a large number of patients with peak height time ranging between 130 s and 260 s, and the number of patients in the premenopausal group was greater than that in the postmenopausal group. There were a large number of patients with early signal enhancement ranging between 100% and 200%, and the number of patients in the premenopausal group was greater than that in the postmenopausal group. In addition, the proportion of patients with ADC value higher than 1.2 × 10^−3^ was the least, and the number of patients in the premenopausal group was greater than that in the postmenopausal group. There were no statistical differences in the types of TIC curves, peak height time, early signal enhancement, and ADC values between the patients in the premenopausal group and the postmenopausal group (*P* > 0.05).

### 3.6. Diagnostic Role of DCE-MRI Examination in Invasive Breast Carcinoma

The comparison of the number of cases with positive and negative invasive breast carcinoma diagnosed by two methods is shown in Figure 7. The sensitivity, specificity, and accuracy of the diagnosis of invasive breast carcinoma by DCE-MRI examination are displayed in Figure 8. Besides, the positive and negative predictive values of the diagnosis of invasive breast carcinoma by DCE-MRI examination are presented in Figure 9. According to pathological examination, there were 128 cases with positive invasive breast carcinoma and 31 with negative one. According to DCE-MRI examination, the number of patients with positive and negative invasive breast carcinoma was 121 and 38, respectively. In addition, the sensitivity, specificity, and accuracy of invasive breast carcinoma by DCE-MRI examination amounted to 91.41%, 87.1%, and 90.57%, respectively. Positive and negative predictive values were 96.69% and 71.05%, respectively.

## 4. Discussion

Breast carcinoma ranks the first among all cancers around the world [12]. In the past few years, breast carcinoma becomes more and more common among youngsters in China [13]. It is a malignant tumor with various morphology, molecular characteristics, clinical courses of disease, and therapeutic response [14]. The prognosis of patients with breast carcinoma is affected by multiple factors, including not only gender, age, lifestyle, and treatment plan but also tumor morphology, pathological levels, lymph node status, immunohistochemical indexes, and gene expression [15, 16].

Fuzzy theory-based can overcome the defects of traditional classification in pixel partition and show excellent fuzziness [17]. Fuzzy theory possesses significant advantage in dealing with uncertain problems [18]. FCM algorithm is an unsupervised image segmentation method widely applied in image segmentation [19, 20], and it is characterized by high sensitivity as well as accuracy and wide application in medical field. Joloudari et al. [21] applied FCM deep neural network (FCM-DNN) in cardiac magnetic resonance CAD imaging dataset and found out that the accuracy of the proposed FCM-DNN model reached 99.91%, which indicated that the model achieved the optimal performance. Praveena and Singh [22] used an analysis FCM algorithm to segment the images of acute lymphocytic leukemia. Besides, they applied the extracted features in deep convolutional neural network for classification. They found out that this method could achieve high accuracy, sensitivity, and specificity. GA-PFCM algorithm was adopted to analyze DCE-MRI features of patients with breast carcinoma, improve image quality, and show good clustering effect. GA-PFCM algorithm could be applied in the processing and segmentation of DCE-MRI images, which had positive promotion values.

To some extent, whether menopause is normal is associated with the occurrence of breast carcinoma. During climacteric period, irregular menstruation occur among women. Hormonal disorders in the body increase the incidence of breast carcinoma [23]. In this research, DCE-MRI imaging features and relevant parameters of patients with breast carcinoma before and after menopause were investigated. According to the research results, the proportion of patients with level 5 breast carcinoma in the postmenopausal group was relatively higher. The proportions of patients with lobular lumps, burrs on lesion edge, and uniformly enhanced lumps in the premenopausal group were higher than those in the postmenopausal group (*P* < 0.05). Besides, there were no statistical differences in TIC curve types, peak height time, early signal enhancement, and ADC values between the premenopausal group and the postmenopausal group (*P* > 0.05). DCE-MRI examination possessed good effects on the assessment of patients' disease before and after menopause.

MRI becomes the current conventional examination, which is superior to other examination methods. It is the preferred diagnostic technique for multiple diseases because of its noninvasiveness, significant pain relief, and high safety [24]. The application of DCE-MRI in tumor evaluation is of great significance, especially in the application of new antitumor targeting drugs and the quantitative functional analysis of then change in membrane permeability of tumors. Besides, DCE-MRI can assess the therapeutic effects of drugs [25]. Therefore, it is of great importance to research the imaging features of DCE-MRI. In the research, the sensitivity, specificity, and accuracy of the diagnosis of invasive breast carcinoma by DCE-MRI examination were discussed. The results demonstrated that there were 128 cases with positive invasive breast carcinoma and 31 with negative one according to pathological examination. In addition, there were 121 cases with positive invasive breast carcinoma and 38 with negative one according to DCE-MRI examination results. The sensitivity, specificity, and accuracy of invasive breast carcinoma by DCE-MRI examination amounted to 91.41%, 87.1%, and 90.57%, respectively. Positive and negative predictive values reached 96.69% and 71.05%, respectively. Based on the above results, it was concluded that DCE-MRI imaging function could be used for the diagnosis of invasive breast carcinoma, which showed guidance significance for the diagnosis and treatment of patients with breast carcinoma.

## 5. Conclusion

The application of GA-PFCM algorithm in the analysis of DCE-MRI image features showed positive significance. The research could provide reference for the diagnosis and prediction pf breast carcinoma with positive clinical significance. The disadvantage of this research was that only the clustering effects of two algorithms were compared. In future, they needed to be compared with other algorithms for further research and demonstration.

## Figures and Tables

**Figure 1:** Specific procedures of GA-PFCM algorithm.

**Figure 2:** Comparison of the number of patients with different levels of breast carcinoma between the two groups.

**Figure 3:** DCE-MRI images of two breast carcinoma patents: (a) lobular lumps; (b) annular enhanced lumps on the edge.

**Figure 4:** Comparison of clustering effects of two algorithms: (a) separation coefficient; (b) separation entropy; (c) firming and separation effects.

**Figure 5:** Comparison of lump features between the two groups during breast DCE-MRI examination: (a) the shape of lumps; (b) burrs on lump edge; (c) lump enhancement.

**Figure 6:** Comparison of DCE-MRI examination parameters of breast between two groups: (a) the types of TIC curves; (b) peak height time; (c) early signal enhancement; (d) ADC values.

**Figure 7:** Comparison of the number of the cases with positive and negative invasive breast carcinoma diagnosed by two methods.

**Figure 8:** Sensitivity, specificity, and accuracy of the diagnosis of invasive breast carcinoma by DCE-MRI examination.

**Figure 9:** Positive and negative predictive values of the diagnosis of invasive breast carcinoma by DCE-MRI examination.

## Data Availability

The data used to support the findings of this study are available from the corresponding author upon request.
